# Investigation and Analysis of the Influence of Vegetative Tracheobronchial Foreign Body on Airflow Field

**DOI:** 10.1155/2022/8930283

**Published:** 2022-04-28

**Authors:** Yudong Bao, Shengqian Qu, Kai Li

**Affiliations:** Key Laboratory of Advanced Manufacturing and Intelligent Technology, Ministry of Education, Harbin University of Science and Technology, Harbin, China

## Abstract

The BSL *k-ω* turbulence model was used to numerically simulate the inspiratory airflow of the airway with foreign bodies using a real CT scan human airway model. The paper selects three foreign bodies with different diameters, three different foreign body positions, and three different breathing intensities, and the FLUENT software is used to perform numerical simulation. This study has found that the increase in the diameter of the foreign body and flow velocity will make the flow structure in the airway more complicated. The airway pressure will increase so that the resistance of breathing will increase, and the shear force will also increase, which hurt the airway. The impact of the foreign body on the left side on the flow structure in the airway is less than that of the foreign body on the right side. The foreign body on the left side causes the pressure drop in the airway to be higher than that on the right side. Moreover, sharp changes in pressure driving force and airway curvature will affect the airflow pattern of the central airway. We concluded that foreign matter has a great influence on the characteristics of the airflow structure, and more research is needed to increase the understanding of the airflow pattern under the condition of foreign matter in the airway, and the research helps doctors avoid the influence of airflow when removing foreign bodies in the airway.

## 1. Introduction

Airway foreign body is a very common respiratory disease in life, which can occur at all ages, especially in children and the elderly. Inhalation of foreign bodies can cause chronic irreversible bronchopulmonary injury, which can seriously lead to sudden cardiac arrest, asphyxia, and even death [1–6]. Among the foreign bodies inhaled, peanuts, soybeans, cashew nuts, and other plant-based foreign bodies accounted for a high proportion. Foreign bodies are mainly located in the right main bronchus, the upper lobe of the right lung, and the left main bronchus [7, 8]. In the process of foreign body removal, the patient needs to be mechanically ventilated, which is a challenge for tracheal surgery. At present, there are few studies on the bronchial airflow environment with foreign bodies, and it is a great difference in ventilation modes during surgery, lacking a unified understanding. In addition, the complexity and uncertainty of airway airflow also increase the difficulty of foreign body forceps. Therefore, this paper investigates the endobronchial airflow environment in the presence of foreign bodies, which can help adjust the mode of mechanical ventilation and prevent the relative motion of the trachea and foreign bodies during ventilation, thus providing theoretical guidance for future automated clamp removal of bronchial foreign bodies.

In recent years, computational fluid dynamics, as a science combining recent fluid dynamics and computer science, has been widely used in the diagnosis and treatment of respiratory diseases, attracting many scholars to study it. In the field of resolving airway model and studying the influence of airflow, Mark et al. used multilayer CT images to construct the original three-dimensional airway geometry and artificially inserted stenoses with different constrictions and lengths; the results showed that the original and smoothed real airway models presented excellent agreement [9]. Fan Y conducted a computational and experimental study of stable inhalation based on a real human airway model and the study showed a good agreement between the numerical and experimental results [10]. Hariprasad et al. studied the pressure and velocity of airflow in the tube during sneezing by using a real human upper breathing model [11]. Shouliang Q compared the velocity and pressure distribution between healthy trachea model and interstitial lung disease model, and the results can be used to judge the influence of disease on mechanical parameters [12]. Shen et al. established the biomechanical models of the trachea and bronchus to study the effects of different breathing modes on airflow characteristics and airway resistance; the results showed that the high-speed region of airflow in the airway was generally distributed in the inner side of the trachea [13]. In the field of airflow numerical simulation, Cui X used large eddy simulation to predict the airflow field in the upper respiratory tract during unsteady respiration, and simulated the airflow in the airway, and found that the airflow structure was greatly influenced by the respiration model [14]. Luo applied the low Reynolds number (LRN) *k-w* turbulence model to numerically simulate the inspiratory flow characteristics of the CT scan human lung model, and finds that the air velocity between the left and right airway is not sensitive to the Reynolds number. In the right airway or left airway, the momentum of airflow is not obvious, and the inlet velocity distribution in the airway not only affects the airflow pattern, but also changes the flow ratio [15]. Singh P et al. numerically simulated three different models of healthy lung and left and right lung tracheal stenosis by using finite element volumetric discrete element method, and obtained the airflow velocity amplitude in the stenosis part [16]. Lin Jiang et al. used large eddy simulation to calculate the gas flow phenomena within a non-regular geometric surface structure, and tracked the motion of particles to obtain the distribution law of secondary airflow velocity for different cross-sections [17].

Currently, many scholars have focused more on the study of the airflow in healthy airways or airways with specific diseases, such as airway stenosis, and less attention is paid to the airflow environment with foreign body in the airway. In addition, the presence of foreign body airway and airway stenosis has a great difference in pathology. Plant foreign body is mainly distributed in the right main bronchus, right upper lobe, left main bronchus, and other places, which are greatly disturbed by airflow. What's more, researchers used different models to study the airway airflow, respectively, but could not get universally applicable conclusions. In this paper, the influence of different diameters and positions of trachea foreign body and different airflow intensities on airway airflow is analyzed, and the airflow characteristics and the force of airflow on foreign body are obtained. The conclusion will not only provide a reference for the diagnosis and mechanical ventilation of tracheal foreign bodies, that can reduce the occurrence of complications, but also provide a theoretical basis for subsequent studies on automated foreign body clamping.

## 2. Materials and Methods

### 2.1. Establishing Airway Model

In this study, the data of an adult male patient were obtained by 256-slice spiral CT scan with a scan thickness of 0.5 mm. The scan data were imported into Mimics21 software for 3D reconstruction to obtain a 3D model of the real trachea (see Figure 1). Since foreign bodies are mainly in the secondary trachea, the model is simplified and the end of the trachea is removed in order to reduce the calculation cost. In Mimics21 software, seven different points were selected from the first two levels of the trachea to measure the reconstructed bronchus. And the measurement data of bronchial diameter, cross-sectional area, and path length were collected, and the geometric parameters of the trachea are shown in Table 1. Koombua found that tissue elasticity only affects the maximum airflow velocity, airflow pressure, and wall shear stress by 2%, 7%, and 6%, respectively, so it is assumed that the geometric model is a rigid body [18]. At the solid boundary of the calculation region, the non-sliding boundary condition was set for the velocity, and the changes of airflow field in the airway of foreign body were discussed under the conditions of three positions, three bodies with different diameters and airflow strengths.

### 2.2. Boundary Conditions

The human respiratory process is a dynamic process, and in the real respiratory process, both the structure of the airway tree and the environment in the human body are very complex, so it is necessary to simplify and assume some parameters in order to complete the calculation. According to whether the entrance velocity of airflow into the upper respiratory tract varies, the respiratory state can be divided into steady and non-steady respiration. This paper mainly considers whether foreign bodies in the airway will have a certain impact on human respiration under three specific states of static, mild, and vigorous exercise. Therefore, the suction rate could be considered a constant value. After referring to the study of lung deposition particles in steady-state respiration, this paper took the average of adult breathing in three states for simulation analysis to better match the real breathing intensity [19].

Assuming that the cycle of human circular breathing is about four seconds, the ratio of exhalation and inhalation time is 1 : 1. According to the study, the flow rate per unit time of normal human breathing is 500 ml/s; the flow rate per unit time of light activity is 1000 ml/s; the flow rate per unit time of vigorous activity is 1500 ml/s [20–22]. Since the majority of plant-based foreign bodies inhaled by humans are peanuts, soybeans, cashews, and so on, their shapes are mostly round or oval. This paper has simplified the foreign bodies as spheres, and selected three different diameters of foreign bodies for analysis, namely, 6 mm, 8 mm, and 10 mm. The locations of vegetative foreign bodies are mainly in the right main bronchus, the upper lobe of the right lung, and the left main bronchus. Therefore, the locations of foreign bodies have been set as location 1, location 2, and location 3. The setting scheme is shown in Table 2.

The fluid is air, so it is necessary to calculate the Mach number and Reynolds number (Re) to determine whether the airflow in the airway can be regarded as an ideal incompressible fluid, which also is helpful to select the fluid calculation model. The calculation formula of Mach number (*Ma*) is as follows:

(1) $$\begin{array}{c} Ma=\frac{v}{c}, \end{array}$$

where *v* is the flow velocity of the inlet fluid; *c* is the local speed of sound, *c* =340 m/s.

When the inlet velocity is 2.1326 m/s, according to the Reynolds number calculation formula (2), the Reynolds number is 2522.24>2300; when the entrance velocity is 4.2653 m/s, the Reynolds number is 5044.599>2300; when the entrance velocity is 6.3978 m/s, the Reynolds number is 7566.721>2300, so the Reynolds numbers are all greater than 2300. Therefore, the Reynolds number is greater than 2300, which is consistent with the turbulent flow of a subsonic fluid.

(2) Re=ρvdμ,

where *ρ* is the density of air, *ρ* =1.225 kg/m^3^; and *d* is the inlet diameter, *d* =17.282 mm; and *μ* is the aerodynamic viscosity, *μ* =1.79 × 10^−5^ Pa‧s.

### 2.3. Governing Equations

From the above analysis, the gas flow in the trachea conforms to the characteristics of subsonic fluid, so the turbulence model is selected. The *BSL k-ω* model combines the *k-ω* model with the *k-ε* model, and retains the precision of the *k-ω* model near the wall. The *k-ε* model is used in the mainstream region, and the results do not depend on the advantages of free flow. Therefore, the calculation results of *BSL k-ω* model are similar to the *k-ω* model in the boundary layer, and gradually transition to the *k-ε* model at the boundary layer to the free surface. Besides, the *BSL k-ω* model requires less iterative steps than the *k-ε* model. When the Reynolds number is large and Re >4000, the results of the *BSL k-ω* model are more accurate, so the *BSL k-ω* turbulence model is selected [23, 24]. The air temperature in the airway is 37°C, so the energy equation can be ignored. The governing equations are as follows:

The continuity equation:

(3) $$\begin{array}{c} \frac{\partial u_{j}}{\partial x_{j}}=0. \end{array}$$

The momentum equation:

(4) $$\begin{array}{c} \frac{\partial u_{i}}{t}+u_{j}\frac{\partial \left(u_{i}\right)}{\partial x_{j}}=-\frac{1}{\rho }\frac{\partial p}{\partial x_{i}}+\frac{u}{p}\frac{\partial^{2}u_{i}}{\partial x_{j}^{2}}, \end{array}$$

where *u*_*j*_ is the 3 coordinate components of the velocity in the coordinate system, *i* = 1,2,3; and *p* is the pressure, and *ρ* and *μ* are the density of the fluid and viscosity coefficient, respectively.

Turbulent kinetic energy *k* equation:

(5) $$\begin{array}{c} \frac{\partial k}{\partial t}-\frac{\tau_{ij}\partial u_{i}}{\partial x_{i}}=\frac{\partial }{\partial x_{j}}\left[\left(v+\sigma_{k}v_{t}\right)\frac{\partial k}{\partial x_{j}}\right]-\beta^{*}\omega k. \end{array}$$

Dissipative power *ω* equation:

(6) $$\begin{array}{c} ⟶\frac{\partial \omega }{\partial t}-\frac{\gamma }{\rho v_{t}}\tau_{ij}\frac{\partial u_{i}}{\partial x_{j}}=\frac{\partial }{\partial x_{j}}\left[\left(v+\sigma_{\omega }v_{t}\right)\frac{\partial \omega }{\partial x_{j}}\right]+2\left(1-F_{i}\right)\sigma_{\omega 2}\frac{1}{\omega }\frac{\partial k}{\partial x_{j}}\frac{\partial \omega }{\partial x_{j}}, \end{array}$$

where *v*_*t*_ is the eddy viscosity; and *σ*_*k*1_, *σ*_*k*2_, *σ*_*ω*1_, and *σ*_*ω*2_ are the Prandtl numbers for *k* and *ω*; *β*_1_, *β*_2_, and *β*∗ are constants, and *k* is von Karman's constant, and *γ*_1_ and *γ*_2_ are constants. The specific parameters in the model are as follows:

(7) $$\begin{array}{c} \begin{array}{c} \sigma_{k1}=0.5,\;\sigma_{k2}=1.0;\;\sigma_{\omega 1}=0.5,\;\sigma_{\omega 2}=0.856;\\ \beta_{1}=0.075,\;\beta_{2}=0.0828;\;\beta^{*}=0.09,\;k=0.41;\\ \gamma_{1}=\frac{\beta_{1}}{\beta^{*}}-\sigma_{\omega 1}\frac{k^{2}}{\sqrt{\beta^{*}}};\;\gamma_{2}=\frac{\beta_{2}}{\beta^{*}}-\sigma_{\omega 2}\frac{k^{2}}{\sqrt{\beta^{*}}}. \end{array} \end{array}$$

The constants for the inner model *ϕ*1 and the outer model *ϕ*2 are given by formula *F*_1_:

(8) $$\begin{array}{c} \phi =F_{1}\phi_{1}+\left(1-F_{1}\right)\phi_{2},\\ F_{1}=\tanh\left(\arg_{1}^{4}\right). \end{array}$$

And arg_1_ is obtained by the following formula:

(9) $$\begin{array}{c} \left|\arg_{1}=\min\right.\left[\max\left(\frac{\sqrt{k}}{0.09\omega y};\frac{500v}{y^{2}\omega }\right);\frac{4\sigma_{\omega 2}k}{{CD}_{k\omega }y^{2}}\right]. \end{array}$$

Besides, *y* is the distance to the wall, which is obtained by the following formula:

(10) $$\begin{array}{c} {CD}_{kw}=\max\left(2\sigma_{\omega 2}\frac{1}{\omega }\frac{\partial k}{\partial x_{j}}\frac{\partial \omega }{\partial x_{j}},10^{-20}\right). \end{array}$$

There the boundary conditions are:

(11) $$\begin{array}{c} k_{\omega }=0,\omega_{\omega }=10\frac{6v}{\beta_{1}{\left(\Delta y\right)}^{2}}. \end{array}$$

## 3. Results and Discussion

A commercial CFD software FLUENT was used to solve the airflow field, and the unstructured tetrahedral mesh was used to divide the trachea model as shown in Figures 2(a) and 2(b). Considering that the airflow would not pass through the foreign body, Boolean calculation was carried out on the trachea and the foreign body, and local mesh refinement was performed for the contact area between the foreign body and the trachea, which could help to improve the accuracy of solving the airflow characteristics near the foreign body. The mesh model of foreign body is shown in Figure 2(c), and the boundary condition of the foreign body was set as the wall condition.

According to the relevant studies on fluid analysis in ducts, grid independence verification was carried out for the trachea foreign body model [25]. Six planes represented in the trachea (planes 2, 3, 4, 5, 7 and exit planes in Figure 3) were selected and the maximum airflow velocity in the six planes was monitored for simulation verification; the results are shown in Figure 4. When the number of elements increases from 216969 to 369886, the line variation of the maximum air velocity of the six planes tends to be consistent, and 216969 elements can be considered to have met the requirements of grid independence. Through the mesh division of the model, a total of 146332, 216969, 288996, and 369886 numerical grids were generated. In addition, the preliminary mesh resolution study showed that the mesh refinement with more than 216,969 elements would not change the airflow velocity distribution in the foreign body airway, the element mass was 0.84, and the pressure change between the inlet and outlet of the model was less than 1%, which could satisfy the subsequent calculation. Similarly, the independence of time step was analyzed under the condition of 216969 elements. The results showed that 0.01 step could satisfy the subsequent calculation.

In addition, it can be seen from Figure 4 that the airflow decreases at the first bifurcation of the trachea and drops sharply near the foreign body. This is because foreign matter obstructs the airway, resulting in reduced airflow into the airway. After the airflow passes through the foreign body, the airflow velocity will increase due to extrusion. At the secondary bifurcation, the airflow velocity will also increase due to the smaller trachea section, which is also in line with the real human environment. Therefore, this can verify the rationality of the model established by us from another aspect.

This article will study the influence of foreign bodies on the airflow in the airway from the airflow velocity, pressure, and shear force. In order to better understand the airflow in the airway under the state of foreign bodies, seven different planes and lines in the tracheal model are selected. Plane1 and line1 are located at the entrance. Plane2 and line2 are located at the tracheal section, and plane3 and line3 are located at the tracheal bifurcation. Plane4 and line4 are located in the central plane of the foreign body at position 1 and pass through the central of mass. Plane 5 and line 5 are located at the right bronchial bifurcation. Plane6 and line6 are located in the left bronchus. Plane7 and line7 are located in the right bronchus, as shown in Figure 3. By establishing different planes, we can more directly observe the influence of foreign bodies on various areas of the trachea. And by observing the velocity contour curve of the straight line, we can see the trend of the influence of foreign bodies on various areas of the trachea. This study can help doctors to diagnose the location of foreign bodies by changes in airflow and pressure, and also enable them to judge the size of shear stress according to the change in airflow, so as to better remove foreign bodies.

### 3.1. The Analysis of Airflow Distribution Cloud Map

The flow rate in the trachea is an important parameter in breathing, which can help doctors judge the intensity of breathing. The diameter of the foreign body is 8 mm, the foreign body is located in position 1 (right airway), the suction velocity is 2.1326 m/s, 4.2653 m/s, 6.3978 m/s, to investigate the effect of airflow on the foreign body at different flow velocities, and the velocity cloud map was obtained as shown in Figure 5. From the figure, we can see that there is no obvious difference between the velocity cloud and streamline plots in plane1, plane2, plane3, and plane5, but all of them are more turbulent than the airflow in the healthy airways. And the airflow vortex in planes 6 and 7 gradually transitioned from two reverse vortices to one vortex, which indicates that the airflow fills faster as the velocity increases and the airflow in the left air duct tends to smooth out.

In order to explore the influence of different foreign body diameters on the airflow characteristics, the gas velocity of seven planes of the trachea during suction is calculated when the foreign body diameter was 6 mm, 8 mm, and 10 mm, the suction velocity is 2.1326 m/s, and the foreign body is located in position 1. The airflow velocity contour and flow line are obtained as shown in Figure 6. It can be seen from the figure that from plane3, the airflow velocity in the healthy right trachea is greater than that in the left trachea, which is due to the short and thick right trachea and the small angle of the long axis of the trachea. With the increase of the diameter of the foreign body, the velocity of the left trachea increased. This is because the blockage of the right trachea aggravated, and more gas entered the left trachea, which increased the burden of the left lung. Plane4 shows that with the increase of the diameter of the foreign body, the plane flow rate increases, which is because the foreign body leads to the decrease of the area of the trachea and the increase of the flow rate in the region where the foreign body exists. Plane6 shows increased right tracheal obstruction and more gas entering left trachea. Figure 6 shows that with the increase of the diameter of the foreign body, the airflow becomes more turbulent. This is because the existence of foreign body makes the area behind the foreign body with relatively low pressure appear, and then forms a vortex, and the airflow becomes more disordered. Therefore, the larger diameter of foreign body will lead to narrowing of the trachea, which will result in a large pressure difference between the left and right trachea, reducing the respiratory strength of the person and leading to asphyxia. At the same time, the increase of foreign body diameter will lead to the increase of the contact area between the body and the airway wall during the operation, which will interfere with mechanical ventilation and is not conducive to the removal of foreign body.

To investigate the influence of the foreign body and the airflow characteristics in the trachea when the foreign body is in different positions in the trachea, the diameter of the foreign body is chosen to be 8 mm, the airflow velocity is 2.1326 m/s, the foreign body is located in position 1, position 2, and position 3, and the velocity cloud diagram is shown in Figure 7. It can be seen from the figure that due to the presence of foreign bodies, the overall airflow in the trachea is disordered, and there is no significant difference between the streamlines in plane1 and plane2. The flow velocity profile changes significantly from plane3. Plane6 shows that the left foreign body affects the right trachea more than the left trachea. Obviously, when the foreign body exists in the right trachea, the airflow has reverse vortex in most planes, and the airflow characteristics are more complicated than the left side, so the foreign body location has a great influence on the airflow characteristics.

Through the analysis of the cloud images of different plane velocities, it can be found that the foreign body has a great influence on the airflow characteristics in the trachea, and the influence on the airflow is different under various conditions. Foreign body in the right airway has a greater impact on airflow environment than on the left. This is due to the distribution of airflow in the lung. The left lung is smaller and narrower than the right lung, resulting in greater airflow resistance, and more air flows to the right lung than the left lung. Therefore, left blockage has a greater impact on the airflow environment in the airway than the right. When the diameter of the inhaled foreign body is too large, or the patient breathes rapidly, the airflow around the air foreign body will be disturbed, thus affecting the patient's life safety, which may affect the process of foreign body removal by the net forceps.

### 3.2. Airflow Analysis in the Main Airway

When the foreign body was located at position 1 and the inspiratory rate was 2.1326 m/s, the foreign body with diameter of 6 mm, 8 mm, and 10 mm was analyzed, and the respiratory curves of line1, line2, and line3 are obtained as shown in Figure 8. The velocity curve of the airflow is similar to a parabolic shape at the velocity section of the respiratory inlet, which becomes partially excessive at line2. The diameter of the airway at line3 becomes larger, and the maximum velocity is lower than line2. The airway in the presence of foreign bodies showed a slight increase in velocity in some areas at line1, with no significant overall difference, and a significant difference at line2. Obviously, in the velocity profile of line2, there is a clear depression in the middle of the curve, and the minimum velocity in the middle is lower than the peak on both sides. Moreover, the larger the diameter of the foreign body, the more severe the central depression. This is because when there is a foreign body in the airway, the foreign body has a certain obstructive effect on the airflow, and the flow rate of airflow to the left bronchus increases, making the flow rate in the area of the foreign body higher, so the flow rate near the right end of the airway increases. As the foreign body diameter increased, the blockage on the right side of the trachea intensified, and the lower the flow rate, the higher the flow rate of the left bronchus. Obviously, strong changes in pressure driving forces and airway curvature can affect airflow patterns in the central airway.

Foreign bodies with a diameter of 8 mm and airflow speed of 2.1326 m/s are selected to analyze foreign bodies at positions 1, 2, and 3, and the velocity contour curves are obtained as shown in Figure 9. It can be seen from the figure that where the velocity dent is the largest, the velocity of the foreign body at position 2 decreases by 5% compared to the healthy airway. When the foreign body is in the left airway, it can be seen from line3 that the velocity of the foreign body in position 2 is 24% lower than that of the healthy airway. And the velocity of foreign body in position 3 is 8% higher than the velocity of healthy airway. At the point where the velocity bulges the most, the velocity of the foreign body in position 2 rises by 30% compared to the healthy airway, the velocity of the foreign body in position 1 rises by 26%, and the velocity of the foreign body in position 3 falls by 12%. Therefore, it can be concluded that the foreign body on the right side has a greater impact on the airflow environment than the left side. This is due to the distribution of airflow in the lungs; the left lung is smaller and narrower than the right, resulting in greater resistance to airflow.

### 3.3. Drawdown Analysis

Airway pressure plays an important role in breathing. When air flows from the high pressure area to the low pressure area, the airway pressure must be lower than atmospheric pressure.  Figure 10 presents the average pressure at selected planes for different inhalation conditions.  Figure 10(a) shows the average pressure of each plane when the inlet velocity is 2.1326 m/s. It can be seen from the figure that when the foreign body diameter is 6 mm, the pressure in each plane increases by about 20%, when the diameter is 8 mm, the pressure increases by about 60%, and when the diameter is 10 mm, the pressure increases by about 150%. The pressure difference between planes 1, 2, and 3 decreases and the pressure drop in the main airway decreases, which indicates that the patient is experiencing difficulty in breathing. This is due to the presence of a foreign body, increasing the pressure in the airway. The larger the diameter of the foreign body, the greater the airway resistance, resulting in more difficulty in breathing. From Figure 10(b), it can be seen that the foreign objects in three different locations make the pressure in planes 1, 2, and 3 increase by more than 30%. Moreover, the left foreign body makes the airway pressure change more intense, and the pressure drop at the left foreign body is higher than the right.  Figure 10(c) shows the average pressure of each plane at different flow velocities. It can be seen from the figure that with the increase of flow velocity, the pressure changes violently, and the pressure increases more than twice in plane1, plane2, and plane3. This indicates that severe breathing can lead to severe changes in airway pressure.

### 3.4. Wall Shear

Figure 11 shows the wall shear at airway when the airflow velocity is 2.1326 m/s, the diameter of the foreign body is 6 mm, 8 mm, and 10 mm, and the position of the foreign body is at location 1.  Figure 10 shows the wall shear at airway when the airflow velocity is 2.1326 m/s, 4.2653 m/s, and 6.3978 m/s, and the diameter of the foreign body is 6 mm. It can be seen from Figure 12 that as the diameter and inlet velocity increase, the wall shear at the airway with the foreign body increases by about 20%. The place where the wall shear is the greatest is the place where the foreign body contacts the wall. This is because the place where the foreign body contacts the airway is narrow, which makes the flow velocity increase around the foreign body. When the flow rate is 4.2653 m/s, the maximum shear force is 170% of 2.1326 m/s. When the flow velocity is 6.3978 m/s, the maximum shear force is 90% higher than that at 4.2653 m/s. The larger the diameter of the foreign body, the narrower the airway, and the airflow velocity is higher, and the wall shearing increase, which aggravates the damage of the foreign body to the airway, especially the area of the foreign body is prone to inflammation, and the increase of the wall shearing will aggravate the inflammation in the airway area.

## 4. Conclusions

This study was conducted to analyze the airflow changes in the presence of foreign bodies in the trachea species by numerical simulation. Based on the 3d reconstructed real airway model, the turbulence model BSL *k-ω* model was selected to study the trachea with foreign body. The results showed that the airflow characteristics in the trachea have great difference. By analyzing the airflow velocity and pressure in the main trachea, this paper obtained the influence of foreign body on the airflow characteristics under different diameters, positions, and respiratory intensity. Finally, this paper compared the finite element results of the foreign body airway, and the healthy airway and obtained the conditions to reduce the airway pressure when removing the foreign body, which can help to avoid the occurrence of airway inflammation and reduce the damage to the airway.

From the results, it can be obtained that the airflow environment in the airway becomes more complex as the foreign body diameter increases, while strong changes in pressure driving force and airway curvature can affect the airflow pattern in the central airway. In addition, the pressure of the main airway will increase with the diameter of the foreign body. When there is a foreign body on one side of the trachea, the flow rate on the other side increases, increasing the burden on the other side. Besides, the presence of foreign bodies in the trachea is easy to form a reverse vortex, so that the airflow in the trachea becomes more chaotic, and the pressure of the trachea will increase, making breathing more difficult. Meanwhile, a larger foreign body will cause an increase in the area of contact with the airway, making the airway subject to a greater shear force, which exacerbates the damage to the airway wall by the foreign body. In particular, the foreign body area is highly inflammable and increased shear will exacerbate the inflammation in the airway area, which increases the patient's pain.

The velocity cloud and flow distribution in the foreign body airway are relatively similar, but it is more turbulent compared to the normal airway airflow environment. The pressure changes dramatically as the flow rate increases, which indicates that the violent breathing can lead to dramatic changes in air pressure in the airway. The higher the airflow velocity, the greater the shear force of the airflow on the airways, thus increasing the risk of inflammation. This is because the airflow will squeeze through both sides of the foreign body when it passes near the foreign body, resulting in the increase of airflow velocity behind the oreign body and disorder. In this case, the foreign body on the gas wall also increased. When the human body does strenuous exercise, such as running and coughing, the body's inspiratory speed increases, thus exacerbating the change of airflow near the foreign body, which will lead to human breathing difficulties. This also reflects the rationality of the calculation model established in this paper.

In summary, foreign bodies have different effects on airway under varied conditions. When the diameter of the foreign body is too large, or the patient breathes rapidly, the airflow in the trachea will be disturbed, thus increasing the pressure in the trachea, which will affect the patient's life safety. In addition, it is found that left side blockage had a greater impact on the airflow environment in the airway than right side. When a foreign body is present in the left airway, the left lung is smaller and narrower than the right lung, which causes greater resistance to airflow. When mechanical ventilation is performed, the airflow enters the right lung, increasing the pressure on the right lung. Therefore, in order to reduce the pain during the removal of foreign bodies, the patient should keep breathing slowly, and the doctor should adjust the mechanical ventilation mode according to the pressure changes in the trachea.

There are still some shortcomings in this paper, such as considering the human respiratory process as a steady-state process, only for the human body several specific inspiratory velocity research, without taking into account the human body in the case of cyclic respiration. The next step of this paper will simulate the real breathing process of human body to explore the impact of foreign bodies on human respiration. The purpose of this study is to explore the airflow characteristics of trachea foreign body in different airflow conditions, different diameters, and different positions of foreign body. The results of this study can help doctors diagnose the position of tracheal foreign body through changes in airflow and determine the shear stress at tracheal according to changes in pressure, so as to help doctors adjust the mode of mechanical ventilation during surgery. This study can make up for the deficiency of the study on the airflow environment when there is foreign body in the airway, and provide a theoretical basis for automatic trachea foreign body extraction in the future.

## Figures and Tables

**Figure 1:** Reconstructed airway models: (a) unsimplified airway model, (b) simplified airway model.

**Figure 2:** Diagram of the trachea and foreign body mesh model. (a) The frontal tracheal mesh model. (b) The side of tracheal mesh model. (c) Foreign body mesh model.

**Figure 3:** Selected lines and planes for velocity profile.

**Figure 4:** Grid independence verification.

**Figure 5:** Velocity contours at different positions for three different airflows velocity.

**Figure 6:** Velocity contours at different positions of the healthy airways and airways with different diameters.

**Figure 7:** Velocity contours at different positions of the healthy airway and foreign bodies of different locations.

**Figure 8:** Velocity profiles for the healthy airway and three foreign bodies of different diameters, at (a) line1, (b) line2, (c) line3.

**Figure 9:** Velocity profiles for the healthy airway and foreign bodies of different locations, at (a) line1, (b) line2, (c) line3.

**Figure 10:** Pressure drops at different positions of airway at (a) different diameters, (b) different positions, and (c) different flow rates.

**Figure 11:** Wall shear for the three lung models at 2.1326 m/s: (a) 6 mm foreign body, (b) 8 mm foreign body, (c) 10 mm foreign body.

**Figure 12:** Wall shear for the three lung models at (a) 2.1326 m/s, (b) 4.2653 m/s, and (c) 6.3978 m/s.

**Table 1:** Statistical table of measurement data at different positions of the trachea.

Location	Diameter (mm)	Cross-sectional area (mm^2^)	Length (mm)
Tracheal position A	19.25	296.62	(OA)48.07
Tracheal position B	19.96	306.95	(AB)50.62
Tracheal position C	22.16	371.92	(BC)44.43
Tracheal position D	15.55	190.68	(CD)18.74
Tracheal position E	10.33	83.66	(DE)25.35
Tracheal position F	13.62	147.22	(CF)25.97

**Table 2:** Simulation scheme.

Condition	Volume flow rate	Location	Foreign body diameter
Data	500	1	6
	1000	2	8
	Shark Bay	3	10

## Data Availability

The data used to support the findings of this study are available from the corresponding author upon request.
